The article "Corporate social responsibility: A key driver of sustainable development in China’s post-COVID economy" was retracted in 2025. Reasons: unreliable results or conclusions; concerns about the authorship; concerns about the article.

# Corporate social responsibility: A key driver of sustainable development in China’s post-COVID economy

**DOI:** 10.1371/journal.pone.0300209

**Published:** 2024-05-31

**Authors:** Muhammad Salman, Yongming Zhu, Saima Kiran, Muhammad Sibt e Ali, Bandeh Ali Talpur, Kazim Raza Talpur, Madeeha Laghari, Samar Raza Talpur

**Affiliations:** 1 School of Management, Zhengzhou University, Henan, China; 2 School of Business, Zhengzhou University, Henan, China; 3 School of Computer Science and Statistics, Trinity College, Dublin, Ireland; 4 Razak Faculty of Technology and Informatics, Universiti Teknologi Malaysia, Kuala Lumpur, Malaysia; 5 School of Public Health, Physiotherapy and Sports Science, University College, Dublin, Ireland; 6 Sukkur IBA University, Sindh, Pakistan; University of Baltistan, PAKISTAN

## Abstract

The first goal of this research was to measure the impact of corporate social responsibility (CSR) on the sustainable development of an organization. However, the second objective examines the moderating influence of government policies, cultural norms, and stakeholder expectations on the relationship between CSR and an organization’s sustainable development. This research primarily focused on the enterprises operating in the energy industry in Beijing. A sample of 498 individuals holding management positions within these enterprises was collected. The study’s results established that CSR significantly influences the sustainable development of firms. Moreover, the results revealed that governmental regulations, cultural norms, and stakeholder expectations play a significant and positive role in moderating the impact of corporate social responsibility on the sustainable development of companies. The results of this study make a valuable contribution to the existing body of literature on CSR and its impact on the sustainable performance of enterprises in China.

## 1. Introduction

COVID-19 has been distributed to the public and private sectors worldwide. The pandemic has left the business sector useless according to its nature and performance. The sustainability of economic affairs for the whole world is disturbed by this pandemic [1]. Similarly, the public and private sector firms in China are also disturbed due to the economic issues faced by the country [2]. The problem becomes critical when the businesses lose the ability to work long-term, but their goals have become to work in the short-term. The short-term workings of businesses have changed the scenario of business performance [3,4]. The credible performance of businesses can be a way forward to improve their performance according to the achievement of organizational goals. Chinese businesses adopt a less productive approach due to less focus on social goals [5]. It is a capitalist approach to run a firm for its profit instead of making profit available to the public for their issues.

The article "Corporate social responsibility: A key driver of sustainable development in China’s post-COVID economy" was retracted in 2025. Reasons: unreliable results or conclusions; concerns about the authorship; concerns about the article.

The energy sector companies’ performance in China has been disturbed due to the attack of COVID-19 [6]. The firm’s performance was disturbed because of the uncertain situation, and working toward achieving social goals was not easy. The durability of any firm’s performance matters a lot, as it has a significant attitude toward its work. The companies in the energy sector lost their share price because of less investment due to business uncertainty [7]. On the other hand, the stakeholders in these companies have an approach to profit generation. This changed the company’s concept and developed negative attitudes to improve performance. Similarly, the management practices of these companies have also decreased due to this research. Indeed, this problem of a firm’s sustainable development is complex, but this practical problem has no solution in the literature.

The existing research on the Chinese energy sector has limitations because the researchers have not focused on sustainable organizational work in COVID-19. Therefore, this practical problem can be improved with supporting literature and recommendations. The existing study by Kong, Antwi‐Adjei [8] reported that corporate social responsibility (CSR) is reliable for the firm performance, but the findings do not support COVID-19. Moreover, research by Vogler and Eisenegger [9] indicated that the sustainability of business performance is critical to achieving organizational goals. Still, there is a lack of research that considers business performance in the context of the recent COVID-19 pandemic. Based on these researchers’ findings, the literature has an open loop. This loop is required to be closed by the findings of this research.

Therefore, the following study is being done to address this gap in the existing body of knowledge. The study objectives are determined based on the research questions. This study aims to investigate the influence of CSR on a company’s sustainable performance. The second study question investigates the moderating influence of government legislation, cultural norms, and stakeholders’ expectations on the relationship between CSR and a firm’s sustainable performance. The scope of this research is confined to both public and private firms operating within China’s energy industry. The findings of this research exhibit a high degree of reliability and have the potential for generalizability, given the characteristics of the sample utilized. This research will contribute to the existing body of literature on CSR and its impact on the sustainable performance of enterprises in China. The present study is structured into several main sections, commencing with an introductory section and a comprehensive literature review. Subsequently, the methodology employed in this research is delineated, followed by an exposition of the data analysis and conclusions. The ensuing section discusses the implications of the study’s results and concludes with a discussion on potential future paths for further investigation.

The article "Corporate social responsibility: A key driver of sustainable development in China’s post-COVID economy" was retracted in 2025. Reasons: unreliable results or conclusions; concerns about the authorship; concerns about the article.

## 2. Review of literature

### 2.1 Legitimacy theory

Legitimacy theory explains that the performance of any firm should be according to the direction of sustainable goals, and it is possible to work for society [10]. Furthermore, this theory highlights that any firm’s long-term survival in society is possible [11]. Based on the foundation of legitimacy theory, organizational work has improved over time. The following research has considered this theory for its framework development. Corporate social responsibility (CSR) measures, such as environmental preservation, ethical labor practices, and community development promotion, can improve a company’s long-term profitability.

Nonetheless, the dynamics of this association are influenced by various moderating factors. These elements include government policies that can reward or enforce corporate social responsibility (CSR) practices. Cultural values also significantly influence society’s expectations and determine the perceived legitimacy of CSR projects. Additionally, stakeholder expectations pressure businesses to match their actions with broader social and environmental goals. The impact of external variables on a firm’s corporate social responsibility (CSR) initiatives is essential in establishing how much CSR contributes to sustainable development, particularly within the context of legitimacy theory.

### 2.2 CSR and firm sustainable development

According to Sarfraz, Ozturk [12], the sustainable development of any firm is possible when the management works strategically to improve its performance. The goals of any firms management are considered appropriate because strategic improvement is possible when fair policies are implemented [13]. Furthermore, any corporation can play a social role when its management has an idea to improve the firm’s performance. Undoubtedly, various organizations have different functions that can influence a firm’s sustainable development, but the responsible role of these firms can play a significant role in the firms performance [14]. Meanwhile, Sarfraz, Ye [15] reported that any firm can have sustainable development when its vision and mission are aligned with its sustainability goals. The advanced working of middle management can support top management’s policies to adopt reliable sustainability goals for firm work [16]. Accordingly, the social aim of any firm should be to enlighten its vision for developing its work for sustainability-related goals. The high-rated sustainable development of any firm can provide a strategic way to advance organizational work [17,18]. In modern countries like the UK, firms have significant policies to work towards achieving sustainability goals. However, organizational management must be productive for advancement [19]. Based on these conceptualizations and theoretical support, the hypothesis below is developed.

The article "Corporate social responsibility: A key driver of sustainable development in China’s post-COVID economy" was retracted in 2025. Reasons: unreliable results or conclusions; concerns about the authorship; concerns about the article.

*H*_*1*_: *CSR has an impact on a firm’s sustainable development*.

### 2.3 Moderating role of government policies

Government policies aim to improve the organization’s working for sustainable development. The advanced work of any firm can be possible when the government has regulations for its working performance [20]. Many firms in the government sector have sustainable working attitudes that could be a way forward to improve organizational management. The reliability of firm performance is based on government policies, and these policies must align with the working approach of the government [21]. When the policies of any government are aligned with advancing sustainability goals, the industrial sectors performance can be improved to support the government [18,22]. The better management of any country is critical when the government is responsible for implementing the regulations related to the social responsibility of businesses [23]. When a business is considered reliable in its working practices, its performance increases over time. Many business institutes work in any country, but the firm performance can only be improved when the management takes serious action [24]. The reliability of organizational improvement and working performance can be a strategic tool for organizational development. The management of businesses is required to have policy implications by considering government regulations [25]. Based on these conceptualizations and theoretical support, the hypothesis below is developed.

*H*_*2*_: *Government policies positively moderate the relationship between CSR and firm sustainable development*.

### 2.4 Moderating role of cultural value*s*

The performance of any organization can be improved when the management is working in a team. The management is responsible for better organizational performance [26]. Organizational goals are achieved when each layer of the management and workforce has a sense of responsibility to work in a team. Organizational management and planning are improved when the diverse team works in collaboration and has a sense of responsibility [27]. The policies can be implemented in any firm based on the decision-making ability and understanding of each other. The performance of firms can be improved when strategic actions are taken for it [28]. The reliability of government performance and organizational working is improved because of the reliable working opportunities [18,29]. The responsible working of an organization is possible with teamwork, and the organizational culture based on collective values can be a significant factor in advancing the performance of any organization [30]. Strategic management in any country can advance its practices, but the reliability of these practices is based on organizational advancement. The organizational working structure for sustainable business development is the best opportunity to achieve organizational goals [31,32]. Based on these conceptualizations and theoretical support, the hypothesis below is developed.

The article "Corporate social responsibility: A key driver of sustainable development in China’s post-COVID economy" was retracted in 2025. Reasons: unreliable results or conclusions; concerns about the authorship; concerns about the article.

*H*_*3*_: *Cultural values positively moderate the relationship between CSR and firm sustainable development*.

### 2.5 Moderating role of stakeholder expectations

Indeed, any firm’s management is responsible for working in the direction of stakeholders. The responsibility of any firm is to work in the direction recommended by the board of directors [33]. However, Sarfraz, Hussain [34] reported that the foremost goal of any firm’s management is to work according to the directors’ guidelines, which should be according to the management’s expectations. Managerial performance can be improved to align the firm with sustainability goals [35,36]. However, it is expected by modern organizations that these organizations should have reliable opportunities to work toward the goals of sustainability. Sustainable working performance is the strategic way to achieve the goals of an organization [37,38]. The stakeholders expect to improve the performance of firms, and the responsibility of any firm management is to work for it. Furthermore, any firm’s stakeholders expect to improve the firm’s performance for the achievement of social goals [39]. The reliability of firm performance and its sustainable advancement can provide a better working opportunity for business [40,41]. Each firm has different goals but must meet the stakeholders’ expectations. Based on these conceptualizations and theoretical support, the hypothesis below is developed, and based on the above literature reviews, the theoretical framework of the study is shown in Fig 1.

*H*_*4*_: *Stakeholder expectations positively moderate the relationship between CSR and firm sustainable development*.

The article "Corporate social responsibility: A key driver of sustainable development in China’s post-COVID economy" was retracted in 2025. Reasons: unreliable results or conclusions; concerns about the authorship; concerns about the article.

**Fig 1:** Theoretical framework.

## 3. Methodology

### 3.1 Measurement and questionnaire development

This study utilized the quantitative design and the scale items were adapted from existing studies. The firm’s sustainable development was measured by indicators adapted from the research by Roxas and Lindsay [42]. The scale items to measure CSR were adapted from the study of Chang [43]. Furthermore, the government policy scale was adopted from the study of Othman, Md. Shaarani [44], to measure the government regulations and incentives for achieving social responsibility. The research methodology flow is presented in Fig 2.

**Fig 2:** Research methodology flow.

Accordingly, the cultural values scale was adapted from the study of Abdullah [45]. Finally, stakeholders’ expectations scale was adapted from the research of Wolff, Parker [46].

### 3.2 Population and sampling technique

The population for this research was the management-level employees of public sector firms operating in China’s energy sector. The capital city was selected for data collection, because it is the hub of government sector companies [3] and the information regarding several companies and employees was collected from the relevant ministry head office upon the personal visit of the authors. As the population was known, this research considered 384 to be the appropriate sample to collect the data recommended by Krejcie and Morgan [47]. Before the data collection, the participants were informed, and written consent was given to the questionnaire. Actual data collection through a self-administered questionnaire started on July 20, 2023, and continued until the end of the month, i.e., July 31, 2023. Furthermore, the cross-sectional data collection technique was applied in this research as this technique is helpful to collect the data when the information is required to be collected at each time. Furthermore, a simple random sampling approach was used to collect the data because the sampling frame for this research was defined, and the population shared a similar trait. The authors distributed 600 questionnaires, and 511 were returned. However, 13 questionnaires with responses were rejected at the preliminary analysis stage. Therefore, the final sample for this research was based on 498 responses, and the data was analyzed using Smart PLS 3. The findings of this research were tested with measurement model assessments and structural model assessments.

## 4. Data analysis and findings

The demographic data is categorized by gender, age groups, and occupation. The majority of respondents are male (45%), with a notable representation of females (25%). In terms of age distribution, the 30–39 age group constitutes the highest percentage (45%), followed by the 40–49 age group (25%). Occupation-wise, managers make up the largest proportion (15%), followed by executives (15%) and supervisors (20%). The data provides insights into the gender and age diversity of management-level employees in the sector, highlighting the dominance of males and the concentration of individuals in the 30–39 age range. Additionally, it underscores the varied occupational roles within the management cadre, with managers being the most prevalent category. Table 1 presents the demographic characteristics of management-level employees in China’s energy sector, based on a sample of 498 respondents.

The article "Corporate social responsibility: A key driver of sustainable development in China’s post-COVID economy" was retracted in 2025. Reasons: unreliable results or conclusions; concerns about the authorship; concerns about the article.

**Table 1:** Demographic information.

**Demographics**	**Gender**	**Age**	**Occupation**
	Male	30–39	Manager
	Female	40–49	Executive
		50–59	Supervisor
		60+	Other
Frequencies	45%	25%	15%

### 4.1 Normality of distribution

This research has tested the collected data to determine the normality of distribution. It is tested to check the data for normality in responses. The findings of skewness and kurtosis determine it. The findings of skewness and kurtosis are essential because they help to understand the normality of distribution. However, the findings of skewness and kurtosis between -2 and +2 are considered acceptable for the normality of distribution [48]. The normality of distribution reported in this research is appropriate and achieves the recommended threshold. The findings are highlighted in Table 2.

**Table 2:** Normality of distribution.

Items	No.	Missing	Mean	Median	Min	Max	Standard Deviation	Excess Kurtosis	Skewness
**CSR1**	1	0	4.107	4	1	5	1.029	0.867	-1.16
**CSR2**	2	0	3.6	4	1	5	1.117	-0.19	-0.59
**CSR3**	3	0	3.985	4	1	5	1.05	0.181	-0.876
**CSR4**	4	0	3.956	4	1	5	1.003	0.155	-0.797
**CSR5**	5	0	3.448	4	1	5	1.143	-0.447	-0.433
**FSD1**	6	0	3.593	4	1	5	1.134	-0.435	-0.514
**FSD2**	7	0	3.596	4	1	5	1.2	-0.514	-0.565
**FSD3**	8	0	4.463	5	1	5	0.929	2.973	-1.855
**FSD4**	9	0	4.211	5	1	5	1.045	0.89	-1.273
**FSD5**	10	0	4.007	4	1	5	1.161	0.517	-1.142
**FSD6**	11	0	4.067	4	1	5	1.172	0.509	-1.185
**GP1**	12	0	3.93	4	1	5	1.148	0.144	-0.955
**GP2**	13	0	4.059	4	1	5	1.124	0.527	-1.14
**GP3**	14	0	4.133	4	1	5	1.074	1.004	-1.28
**GP4**	15	0	3.774	4	1	5	1.267	-0.383	-0.788
**GP5**	16	0	3.667	4	1	5	1.205	-0.461	-0.639
**CV1**	17	0	3.993	4	1	5	1.054	0.35	-0.939
**CV2**	18	0	4.056	4	1	5	0.997	0.49	-0.97
**CV3**	19	0	4.015	4	1	5	1.029	0.651	-1.014
**CV4**	20	0	4.056	4	1	5	1.051	0.67	-1.094
**CV5**	21	0	3.974	4	1	5	1.117	0.475	-1.039
**SE1**	22	0	3.8	4	1	5	1.111	0.083	-0.82
**SE2**	23	0	3.881	4	1	5	1.119	0.338	-0.96
**SE3**	24	0	4.059	4	1	5	1.144	0.683	-1.193
**SE4**	25	0	3.726	4	1	5	1.105	-0.161	-0.666
**SE5**	26	0	3.815	4	1	5	1.113	-0.066	-0.794

The article "Corporate social responsibility: A key driver of sustainable development in China’s post-COVID economy" was retracted in 2025. Reasons: unreliable results or conclusions; concerns about the authorship; concerns about the article.

### 4.2 Items reliability

The reliability of individual items used to measure different constructs is tested at this stage. The validity of these items is tested with the findings of factor loadings. The factor loading threshold of 0.60 is considered significant for the reliability of the individual items, and the items loaded below this threshold aren’t considered appropriate. In this case, the items loaded below 0.60 should be deleted [49]. The reliability of individual items is reported in Table 3 and Fig 3.

**Fig 3:** Individual items reliability. FSD = Firm’ Sustainable Development, CSR = Corporate Social Responsibility, CV = Cultural Values, GP = Government Policies, and SE = Stakeholders’ Expectations.

**Table 3:** Individual items reliability.

Items	CSR	CV	FSD	GP	SE
**CSR1**	0.685				
**CSR2**	0.68				
**CSR3**	0.826				
**CSR4**	0.862				
**CSR5**	0.741				
**CV1**		0.874			
**CV2**		0.874			
**CV3**		0.848			
**CV4**		0.909			
**CV5**		0.859			
**FSD1**			0.628		
**FSD2**			0.68		
**FSD3**			0.657		
**FSD4**			0.851		
**FSD5**			0.853		
**FSD6**			0.822		
**GP1**				0.871	
**GP2**				0.876	
**GP3**				0.834	
**GP4**				0.854	
**GP5**				0.632	
**SE1**					0.851
**SE2**					0.894
**SE3**					0.775
**SE4**					0.667
**SE5**					0.645

### 4.3 Measurement model assessment

#### 4.3.1 Convergent validity

The convergent validity of this research is tested with the findings of composite reliability and average variance extraction. The composite reliability is used to test the internal consistency between the constructs. Furthermore, the findings of composite reliability of more than 0.70 are acceptable for significant convergent validity [50]. Similarly, the results of average variance extraction greater than 0.50 are accepted for significant variance between data [51]. The results reported in Table 4 confirm that this research has achieved convergent validity.

**Table 4:** Convergent validity.

Items	Composite Reliability	Average Variance Extracted (AVE)
**CSR**	0.873	0.581
**CV**	0.941	0.762
**FSD**	0.886	0.569
**GP**	0.909	0.67
**SE**	0.855	0.551

#### 4.3.2 Discriminant validity

The findings of discriminant validity are tested in this research to determine the multicollinearity issues between the items used to measure the relationship between different variables. This research has considered the Heteritrait-Monotrait (HTMT) method for the determination of discriminant validity. The discriminant validity of this test is acceptable when the findings of the HTMT matrix are less than 0.90 [52]. The statistical data reported in Table 5 and Fig 4 confirmed the discriminant validity achieved in this research.

The article "Corporate social responsibility: A key driver of sustainable development in China’s post-COVID economy" was retracted in 2025. Reasons: unreliable results or conclusions; concerns about the authorship; concerns about the article.

**Fig 4:** HTMT Values. FSD = Firm’ Sustainable Development, CSR = Corporate Social Responsibility, CV = Cultural Values, GP = Government Policies, and SE = Stakeholders’ Expectations.

**Table 5:** HTMT.

Items	CSR	CV	FSD	GP	SE
**CSR**					
**CV**	0.649				
**FSD**	0.877	0.621			
**GP**	0.848	0.751	0.794		
**SE**	0.746	0.745	0.698	0.804	

#### 4.3.3. Common method bias

The findings of the variance inflation factor determine the standard method bias. This is also determined to check the collinearity issues among the data. The results of a variance inflation factor less than 3.3 are considered significant for no collinearity issues among the research data [53]. The results are significant and reported in Table 6.

**Table 6:** Common method bias.

	CSR	CV	FSD	GP	SE
**CSR**			2.155		
**CV**			2.598		
**FSD**					
**GP**			2.551		
**SE**			2.746		

### 4.4 Structural model assessment

#### 4.1 Path findings

The findings of the structural model assessment, as shown in Fig 5, are used to test the relationship between the hypotheses. The recommendations of Ramayah, Cheah [54] were followed to check the findings of paths. The T-statistics of more than 1.96 and p-values of less than 0.50 are considered appropriate for the significant hypothesis. The data for this research is reported in Table 7. The first hypothesis’s findings reported that CSR’s impact is positively accepted on a firm’s sustainable development, and hypothesis 1 is accepted. Furthermore, the data reported that the second hypothesis is accepted, and the moderating impact of government policies is significant between CSR and firm’ sustainable development. Likewise, the data reported that the third hypothesis is accepted, and the moderating impact of cultural values is significant between CSR and firm’ sustainable development. Finally, the data reported that the last hypothesis is accepted, and the moderating impact of stakeholders’ expectations is significant between CSR and the firm’s sustainable development.

**Fig 5:** Structural model assessment.

**Table 7:** Path findings.

Path Findings	Original Sample	Standard Deviation	T Statistics	P Values
CSR -> FSD	0.270	0.054	5.026	0
Moderating Effect of Government Policies -> FSD	0.612	0.066	9.298	0
Moderating Effect of Cultural Values -> FSD	0.139	0.028	4.964	0
Moderating Effect of Stakeholders’ Policy -> FSD	0.248	0.031	8.000	0

### 4.2 Moderating effects

The moderating relationships developed in this research are significant. The findings of moderating relationships improved the inconsistency in the existing relationship. The research findings of hypothesis 2 confirmed that the moderation of government policies strengthens the relationship between CSR and firm’ sustainable development. The results reported that a higher rate of government policies could improve the positive relationship between CSR and firm’ sustainable development. The statistical findings are shown in Fig 6.

The article "Corporate social responsibility: A key driver of sustainable development in China’s post-COVID economy" was retracted in 2025. Reasons: unreliable results or conclusions; concerns about the authorship; concerns about the article.

**Fig 6:** Moderating effect of government policies. FSD = Firm’ Sustainable Development, CSR = Corporate Social Responsibility, and GP = Government Policies.

Furthermore, the research findings of hypothesis 3 confirmed that the moderation of cultural values strengthens the relationship between CSR and a firm’s sustainable development. The results reported that a higher rate of cultural values could improve the positive relationship between CSR and a firm’s sustainable development. The statistical findings are shown in Fig 7.

**Fig 7:** Moderating effect of cultural values. FSD = Firm’ Sustainable Development, CSR = Corporate Social Responsibility, and CV = Cultural Values.

The research findings of hypothesis 4 confirmed that moderating stakeholders’ expectations strengthens the relationship between CSR and a firm’s sustainable development. The results reported that the higher rate of stakeholders’ expectations could improve the positive relationship between CSR and the firm’s sustainable development. The statistical findings are shown in Fig 8.

**Fig 8:** Moderating effect of stakeholders’ expectations. FSD = Firm’ Sustainable Development, CSR = Corporate Social Responsibility, and SE = Stakeholders’ Expectations.

### 4.3 Coefficient of determination, predictive relevance, and effect size

The findings of the coefficient of determination are checked to determine the variance between research findings. The findings reported that the variance between research models is 70%. Furthermore, the predictive relevance is determined to confirm the predictive ability of the independent variable on the dependent variable. The findings of predictive relevance greater than 0 are accepted [55]. However, this research reported significant predictive relevance for this research. Furthermore, the effect size is also determined in this research. The effect size is tested to determine the effect of different variables on the dependent variable. The effect size values of 0.02, 0.15, and 0.35 are small, medium, and large effect sizes, respectively [56]. The data highlighted that the independent and moderating variables significantly affect a firm’s sustainable development. The findings are reported in Table 8.

**Table 8:** Coefficient of determination, predictive relevance and effect size.

**Coefficient of Determination**			
**Variables**	**R Square**	**R Square Adjusted**	
**FSD**	0.713	0.709	
**Effect Size**			
**Variables**	**FSD**		
**CSR**	0.128		
**CV**	0.002		
**GP**	0.534		
**SE**	0.001		
**Predictive Relevance**			
**Variables**	**SSO**	**SSE**	
**CSR**	1350	1350	Q^2^ (= 1-SSE/SSO)
**CV**	1350	1350	
**FSD**	1620	985.273	
**GP**	1350	1350	0.392
**SE**	1350	1350	

The article "Corporate social responsibility: A key driver of sustainable development in China’s post-COVID economy" was retracted in 2025. Reasons: unreliable results or conclusions; concerns about the authorship; concerns about the article.

## 5. Discussion of findings

The findings of this research are tested with statistical evidence to confirm the theoretically developed relationships. The objective of this research is achieved as the findings have answered the research questions. Firstly, this research has determined the findings of the first hypothesis, and the results are significant. The first hypothesis path findings confirm that the impact of CSR is significant on a firm’s sustainable development. This relationship was developed theoretically, but the empirical results also supported the theoretically developed relationship between CSR and firm’ sustainable development. However, the results of this hypothesis are theoretically supported by the findings of existing studies. According to Li and Yang [23], middle management’s innovative operations can support top management’s decisions to adopt trustworthy sustainability objectives for business operations. Therefore, each company’s social goal should be to clarify its vision for advancing its projects to achieve sustainability-related objectives. According to Liu, Gao [37], any company’s highly regarded sustainable development might offer a tactical means of enhancing organizational performance. Businesses in developed nations like the UK have essential policies in place to work towards achieving sustainability goals. According to Khuong and Anh [26], organizational management is necessary to contribute positively to organizational progress. Any company can grow sustainably if the management actively works to raise performance. According to Alwakid, Aparicio [27], the objectives of any firm’s management are seen as proper because when just policies are put into place, strategic improvement is attainable. Additionally, any organization can play a social role if its management suggests enhancing the company’s functioning. According to Robaina and Madaleno [24], different organizations serve various purposes that can affect a company’s ability to develop sustainably. Still, these organizations’ socially responsible actions can significantly impact how well a company performs. According to Chouaibi, Rossi [57], any company can achieve sustainable development if its vision and objectives align with sustainability principles.

Furthermore, this research has determined the findings of the second hypothesis, and the results are significant. The second hypothesis path findings confirm that the moderating impact of government policies positively influences and strengthens the relationship between CSR and firm’ sustainable development. No doubt, this relationship was developed theoretically, but the empirical results also supported the theoretically developed moderating relationship of government policies between CSR and firm’ sustainable development. Still, the results of this hypothesis are theoretically supported by the findings of existing studies. According to Phan, Tran [31], although the government is charged with enforcing laws relating to the social responsibility of corporations, more excellent management of the nation is essential. When a company is regarded as trustworthy in its operations, its performance improves. According to Javeed, Teh [30], numerous business schools operate in every nation, but the company’s performance can only be raised when the management makes genuine efforts. An effective strategy for organizational growth can be found in the consistency of organizational progress and working performance. According to Wu, Monfort [20], businesses must evaluate how government rules may affect their management decisions. Government policies are responsible for enhancing how organizations function for sustainable development. According to Lusiana, Haat [35], advanced working is conceivable when the government establishes regulations for how well a corporation performs its function. Many businesses in the public sector have a long-term outlook on work that may pave the way for future advancements in organizational administration. According to Oware and Mallikarjunappa [21], government policies, which must be consistent with how the government conducts business, are the foundation for the dependability of corporate performance. Meanwhile, Rossi, Chouaibi [58] reported in the literature that the performance of the industrial sector can be enhanced to assist any government whose policies align with achieving sustainability goals.

The article "Corporate social responsibility: A key driver of sustainable development in China’s post-COVID economy" was retracted in 2025. Reasons: unreliable results or conclusions; concerns about the authorship; concerns about the article.

Accordingly, this research has determined the findings of the third hypothesis, and the results are significant. The third hypothesis path findings confirm that the moderating impact of cultural value positively influences and strengthens the relationship between CSR and a firm’s sustainable development. Although this relationship was developed theoretically, the empirical results Interestingly, the results of this hypothesis are theoretically supported by the findings of existing studies. According to ElAlfy, Palaschuk [59], organizational and government performance are more reliable when considering dependable employment possibilities. Teamwork makes it feasible for an organization to operate responsibly, and an organizational culture built on shared values can significantly improve any organization’s performance. According to Ndubisi, Zhai [19], any nation can advance strategic management techniques, but the dependability of these techniques depends on organizational development. The most effective way to accomplish organizational objectives is through the functioning structure of the organization for sustainable company development. According to Pizzi, Del Baldo [60], performance in any company can be raised when the management collaborates as a team. A significant duty of the management is to improve the organization’s performance. According to Amorelli and García‐Sánchez [28], achieving organizational goals depends on each management level and the workforce feeling accountable for cooperating as a team. Organizational management and planning are improved when the heterogeneous team collaborates and feels responsible for their work. According to Lopez [17], any firm can adopt policies depending on the ability to make decisions and the level of interpersonal understanding. According to Chouaibi, Rossi [61], when strategic initiatives are implemented, businesses can perform better by employing CSR practices.

Finally, this research has determined the findings of the last hypothesis, and the results are significant. The fourth hypothesis path findings confirm that the moderating impact of stakeholders’ expectations positively influences and strengthens the relationship between CSR and firm’ sustainable development. Moreover, this relationship was developed theoretically, but the empirical results also supported the theoretically developed moderating relationship of stakeholders’ expectations between CSR and the firm’s sustainable development. Yet, the results of this hypothesis are theoretically supported by the findings of existing studies. According to Avotra, Chenyun [13], sustainable working efficiency is the most effective strategy for achieving an organization’s objectives. The stakeholders’ desired outcome is improving business performance, and any firm administration must work towards this goal. According to Ang, Shao [25], stakeholders in any company expect the company to perform better to meet social goals. Better employment opportunities for a company may be made possible by the consistency of firm performance and its advancement in operating. According to Wang, Peng [39], while each company undoubtedly has different objectives, all of them must live up to the expectations of its stakeholders. The management of any company must work in the stated direction of the stakeholders. According to Dhar, Sarkar [14], companies must follow the board of directors’ suggestions to succeed. Working within the directors’ rules and ensuring they meet management standards are the top priorities for each company’s management. According to Hu, Qiu [33], boosting managerial effectiveness and bringing the company closer to the sustainability objectives is possible.

The article "Corporate social responsibility: A key driver of sustainable development in China’s post-COVID economy" was retracted in 2025. Reasons: unreliable results or conclusions; concerns about the authorship; concerns about the article.

## 6. Conclusion

The objective of this study was to examine the effects of Corporate Social Responsibility (CSR) on a company’s sustainable growth, while also considering the moderating factors of government policies, cultural values, and stakeholders’ expectations. The results validate the theoretical frameworks formulated for each hypothesis by confirming substantial associations and offering empirical substantiation. The collective discoveries emphasize the complex and diverse factors that impact a company’s long-term growth, with corporate social responsibility (CSR) serving as a key catalyst. Furthermore, the study highlights the interdependence of government policies, cultural values, and stakeholders’ expectations in determining the influence of CSR on sustainable development. These observations contribute to the wider comprehension of organizational dynamics, offering practical implications for companies seeking to improve their sustainable development. Understanding the impact of corporate social responsibility (CSR), as well as the ways in which external factors can moderate this impact, can help inform strategic decision-making and promote a comprehensive approach to corporate sustainability. In summary, this research not only confirms the theoretical links between CSR and sustainable development, but also emphasizes the significance of external factors in shaping and strengthening these connections. The findings provide valuable insights for businesses, policymakers, and researchers who are interested in promoting sustainable practices in the corporate sector.

## 7. Implications

This research has contributed to the literature and body of knowledge. Similarly, the practical importance of this research is reliable for the practices to adopt CSR as a critical driver for sustainable development in the Chinese economy in the post-pandemic scenario. This research closed a loop in the literature and introduced the moderating variables that improved the knowledge. The existing literature before this research showed inconsistency in the relationship between CSR and firms’ sustainable development. However, this research reported that this inconsistent relationship could be positively strengthened with the moderating role of government policies. This means that when government policies are implemented in organizations, CSR would be fairly implemented for the firm’s sustainable development. Furthermore, this research reported that this inconsistent relationship could be positively strengthened with the moderating role of cultural values. This means that when cultural values are fairly implemented in organizations, CSR would be fairly implemented for the firm’s sustainable development. Finally, this research reported that this inconsistent relationship could be positively strengthened with the moderating role of stakeholders’ expectations. This means that when government policies are pretty implemented in organizations, CSR is fairly implemented for the firm’s sustainable development.

The article "Corporate social responsibility: A key driver of sustainable development in China’s post-COVID economy" was retracted in 2025. Reasons: unreliable results or conclusions; concerns about the authorship; concerns about the article.

The practical implications of this research are noteworthy, as it underscores the positive impact on employee performance when government policies are effectively implemented within organizations. Moreover, the managerial staff would adhere to governmental regulations about sustainability objectives, facilitating the integration of CSR initiatives to attain sustainability within the organizational framework. Moreover, this study posited that senior-level executives are responsible for formulating the vision and goal of the organization in alignment with governmental objectives. Additionally, this study emphasized the need for cultural values about collective collaboration among individuals from varied backgrounds to promote organizational sustainability. The use of fair working policies to meet sustainability goals has the potential to enhance cultural values and government performance. Implementing government policies by management is crucial for enhancing organizational operations and fostering the long-term sustainability of the enterprise. Consequently, company management must align their actions with stakeholders’ expectations, particularly regarding financial considerations, to pursue sustainability objectives and ensure long-term viability effectively. The findings of this study have the potential to be applied broadly to enhance the operational effectiveness of any organization through the implementation of CSR practices.

### 7.1 Limitations and future directions

Although this research has closed a loop in the literature with its findings, the study has developed reliable findings. However, there are some limitations of this research. Firstly, this research has introduced the moderating variables to determine which variable can significantly reduce inconsistency between the relationship of CSR and firm’ sustainable development. This is the limitation of this research because there could be significant mediators that could mediate the relationship between CSR and a firm’s sustainable development. Furthermore, this research’s findings have limitations as it only collected data from middle-level management. Future studies are motivated to collect customer data to understand the importance of these significant findings. Accordingly, this research has considered the quantitative data for findings, but bibliographic research is needed to determine the status of the research and thematic analysis for future research recommendations. By following these directions, scholars can contribute to the literature with significant findings that are reliable for practical work.
